# The Association of Psychosocial Manifestations and Quality of Life With Inflammatory Markers in SARS-CoV-2 Patients: A Study From a Dedicated COVID-19 Tertiary Care Hospital

**DOI:** 10.7759/cureus.42341

**Published:** 2023-07-23

**Authors:** Kuldeep Kumar, Shruti Srivastava, Akshay Meena, Rajnish K Avasthi, Bineeta Kashyap

**Affiliations:** 1 Department of Medicine, University College of Medical Sciences and Guru Teg Bahadur Hospital, New Delhi, IND; 2 Department of Psychiatry, University College of Medical Sciences and Guru Teg Bahadur Hospital, New Delhi, IND; 3 Department of Microbiology, University College of Medical Sciences and Guru Teg Bahadur Hospital, New Delhi, IND

**Keywords:** mental well-being, depression anxiety and stress scale (dass-21), who quality of life brief version (whoqol-bref), second wave of covid-19 pandemic, quality of life, inflammatory markers, covid-19, sars-cov-2

## Abstract

Aim: The second wave of the coronavirus disease 2019 (COVID-19) pandemic adversely affected an individual's physical and psychological well-being. Events such as nationwide lockdown, isolation, social distancing, loss of jobs, and mortality among close contacts and the neighborhood had a dreadful impact on the psychological well-being of the population. At the time of conducting the present study, limited literature was available on the psychosocial manifestations of severe acute respiratory syndrome coronavirus 2 (SARS-CoV-2) infection in the Indian population. Hence, the present study was conducted to find out the association between depression, anxiety, stress, and quality of life with inflammatory markers such as C-reactive protein (CRP), interleukin-6 (IL-6), D-dimer, serum ferritin, procalcitonin (PCT) in SARS-CoV-2 patients during admission and follow-up in a tertiary care hospital.

Methods: This was an observational analytical study conducted during the second wave of the SARS-CoV-2 pandemic at a designated COVID-19 tertiary care hospital in New Delhi, India. Guidelines provided by the Ministry of Health and Family Welfare; the Government of India, were used for deciding hospital admissions. Sixty patients, confirmed positive by reverse transcriptase-polymerase chain reaction (RT-PCR) for SARS-CoV-2, aged 18-60 years, were recruited for this study. All study subjects were screened by a rating scale for which the Hindi version of the 21-item Depression, Anxiety, and Stress Scale (DASS-21) questionnaire was employed, and the Hindi version of the 26-item World Health Organization Quality of Life Brief Version (WHOQOL-BREF) was used to assess the quality of life. Special investigations like CRP, IL-6, D-dimer, serum ferritin, and PCT were sent on day one of admission.

Results: The prevalence of depression, anxiety, and stress was 63.3%, 85%, and 26.7%, respectively. The mean D-dimer level was found to be 957.32 ± 650.91 ng/ml, mean pro-calcitonin level was 1.04 ± 1.47 ng/ml, mean serum ferritin level was 722.24 ± 486.75 µg/L, mean CRP level was 65.36 ± 35.12 mg/L, and mean IL-6 level was 62.79 ± 49.05 pg/ml. The average score for the physical domain of the WHOQOL-BREF on days 7, 14, and 28 were 66.23, 77.43, and 82.18, respectively. The average score for the psychological domain on days 7, 14, and 28 were 73.93, 78.33, and 86.21, respectively. The average score for social domain on days 7, 14, and 28 were 82.63, 86.38, and 89.73, respectively. The average score for the environmental domain on days 7, 14, and 28 were 78.33, 88.78, and 90.98, respectively. The prevalence and severity of depression were significantly associated with D-dimer, CRP, ferritin, PCT, and Interleukin-6 (p<0.05). The prevalence and severity of anxiety were significantly associated with PCT, IL-6, and CRP (p<0.05).

Conclusion: SARS-CoV-2 infection adversely affected our study population's mental well-being. An increased prevalence of psychosocial manifestations like depression, anxiety, and stress was noted in participants. We also concluded that increased levels of inflammatory markers (CRP, IL-6, PCT, D-dimer, and serum ferritin) were associated with increased prevalence of psychiatric manifestations like depression.

## Introduction

The World Health Organization (WHO) designated the severe acute respiratory syndrome coronavirus 2 (SARS-CoV-2) infection as a public health emergency of international concern on January 30, 2020, and declared the outbreak a pandemic on March 11, 2020. By August 2021, the virus had caused more than 200 million confirmed cases and more than 4.3 million deaths worldwide [1].

The second wave of the coronavirus disease 2019 (COVID-19) pandemic was more dreadful than its preceding wave. It lasted from March 2021 to June 2021. By May 8, 2021, India had reported around 26.4 million confirmed SARS-CoV-2 cases and more than 2.74 million deaths [2].

The onset of disease manifestation usually begins within four to five days after exposure. Symptoms include cough, fever, myalgia, headache, dyspnea, sore throat, gastrointestinal symptoms like nausea, vomiting, or diarrhea, dysgeusia, and anosmia [3]. Apart from the typical signs and symptoms of SARS-CoV-2, psychiatric manifestations like depression, stress, anxiety, and poor quality of life have also been reported in SARS-CoV-2 patients globally. Similar psychiatric manifestations were also reported in previous coronavirus outbreaks like severe acute respiratory syndrome (SARS) and Middle East respiratory syndrome (MERS) [3].

Preventive measures for COVID-19 like social distancing, social isolation, quarantine, limiting travel, and working from home had certain negative effects on the mental well-being and health of individuals [4]. They may lead to psychiatric manifestations like depression, stress, anxiety, and poor quality of social life among the patients. Risk factors for developing depression, anxiety, and stress in SARS-CoV-2 may include pre-existing psychiatric illnesses, previously diagnosed malignancy, chronic illness, present or past history of substance abuse, isolated lifestyle, lower education levels, and loss of livelihood [5].

Severe SARS-CoV-2 infection is characterized by the uncontrolled release of pro-inflammatory cytokines, which is known as a cytokine storm. When cytokines and chemokines spill in circulation, this leads to a systemic cytokine storm which can further result in multi-organ dysfunction syndrome (MODS). Cytokine storm is associated with both the inflammatory process as well as suppressing the levels of dopamine and serotonin in the brain, which causes low mood, stress, and anxiety [6].

SARS-CoV-2 causes the downregulation of angiotensin-converting enzyme 2 (ACE-2) receptors. As a result, angiotensin 2 increases in the brain. Angiotensin 2 acts on angiotensinT1 receptors and increases pro-oxidative stress and inflammation in the brain, which leads to the depletion of brain-derived natriuretic factor (BDNF) in the brain. Low levels of BDNF are suggested to be associated with low mood and depression. Bouças et al. showed a positive association between depression and inflammatory processes [7].

The present study aimed to explore the prevalence of depressive symptoms, anxiety, and stress in SARS-CoV-2 patients admitted to a designated COVID-19 tertiary care hospital and the correlation between psychiatric comorbidities and inflammatory markers like C-reactive protein (CRP), interleukin-6 (IL-6), D-dimer, serum ferritin, and procalcitonin (PCT). This study also investigated the quality of life of individuals suffering from SARS-CoV-2 infection (on day 7 of admission in the hospital, on day 14, and on day 28 after discharge).

## Materials and methods

Study design and population

This study was an observational analytical study conducted by the departments of Medicine, Psychiatry, and Microbiology of the University College of Medical Sciences, New Delhi, India, on SARS-CoV-2 patients admitted to a designated COVID-19 tertiary care hospital, Guru Teg Bahadur Hospital, New Delhi, India, during the second wave of the COVID-19 pandemic. The study was approved by the Institutional Ethics Committee - Human Research, University College of Medical Sciences (IECHR/2020/PG/46/38 dated December 2, 2020).

Sample size

To the best of the knowledge of the authors, there was no study on the psychosocial manifestations and quality of life of SARS-CoV-2 patients in the Indian population at the time of conducting the present study. Therefore, to get the maximum sample size, the estimated prevalence of psychiatric morbidity in COVID-19 was assumed to be 50%. For an estimated prevalence of 50%, considering absolute error as 10%, and confidence interval as 95%, the sample size was calculated using the following formula:

 n = Z^2^ x (pq/e^2^)

 n = 1.96^2^ x (50x50/10^2^) = 96

where, Z is a constant with a value of 1.96 at a confidence interval of 95%, p is prevalence, and e is permissible error.

Taking into consideration the financial constraint, and the research being a time-bound work during the COVID-19 pandemic, it was decided to take a sample size of 60.

Data collection and evaluation

Guidelines provided by the Ministry of Health and Family Welfare, Government of India, were used for deciding hospital admissions, which are as follows: (i) Mild: Upper respiratory symptoms and/or fever without shortness of breath or hypoxia; (ii) Moderate: Patients having respiratory rate > 24/minute or oxygen saturation> 90% but < 93% on room air; and (iii) Severe: Patients having respiratory rate > 30/minute or oxygen saturation < 90% on room air. SARS-CoV-2 patients in the mild category required only home isolation and care, those in the moderate category were admitted to wards, while patients in the severe category required intensive care unit (ICU) admission [8].

Sixty patients, confirmed positive by reverse transcriptase-polymerase chain reaction (RT-PCR) for SARS-CoV-2, meeting the inclusion criteria, and aged 18-60 years were recruited for the study. Detailed clinical history, examination, and investigations were carried out as per the case record sheet (chief complaints, history of presenting complaints, general physical examination, systemic examination, mental state examination, and routine investigations). Detailed psychiatric evaluation including detailed psychiatric history taking and mental state examination of all study subjects was done after the initial stabilization of the patient. Those patients who had SpO2 >95% over the last 24 hours were included.

Special investigations like CRP, IL-6, D-dimer, ferritin, and PCT were sent on day one of admission. CRP levels were estimated using the turbidimetric latex-enhanced immunoassay method. IL-6 levels were estimated by commercially available enzyme-linked immunosorbent assay (ELISA), Invitrogen Human IL-6 High Sensitivity ELISA Kit (Thermo Fisher Scientific Inc., Waltham, Massachusetts, United States), as per the manufacturer’s instructions.

All study subjects were screened by a rating scale for which the Hindi version of the Depression, Anxiety, and Stress Scale (DASS-21) questionnaire was employed. DASS 21 is a 21-item questionnaire. The questions are further divided into three self-reporting scales with seven questions each. Depression, Anxiety, and Stress levels were measured and classified into normal, mild, moderate, severe, and extremely severe categories [9]. For those patients who were positive on screening, a psychiatry referral was sent and in consultation with a qualified psychiatrist, psychiatric evaluation was done. Psychiatric diagnosis was confirmed by a trained psychiatrist and appropriate psychiatric interventions were done. The non-pharmacological intervention included specially tailored tele-counseling therapy sessions for COVID-19 patients, which were carried out for all study subjects by experienced psychiatrists. 

The Hindi version of the World Health Organization Quality of Life Brief Version (WHOQOL-BREF) was used to assess the quality of life in recovered SARS-CoV-2 patients. WHOQOL-Bref is a 26-item questionnaire with four domains: Physical, Psychological, Social, and Environmental. Scores of each domain were measured separately. The first assessment was done on day seven of admission. A re-evaluation of the quality of life parameters was done on day 14 and day 28 from the date of discharge [10].

Statistical analysis

The data obtained from the study was entered and cleaned in Microsoft Excel (Microsoft Corporation, Redmond, Washington, United States). Data were analyzed using IBM SPSS Statistics for Windows, Version 20.0 (Released 2011; IBM Corp., Armonk, New York, United States). The categorical variables were expressed in percentages and quantitative variables as mean ± SD. The test of significance for categorical variables was the chi-square test (Fisher's exact test if needed), and for quantitative variables, the independent and paired student t-test/ANOVA test. Correlation and regression analysis was done to study the association between inflammatory biomarkers (CRP, IL-6, D-dimer, ferritin, PCT) and psychiatric morbidities (depression, anxiety, and stress). P-value <0.05 was considered significant.

## Results

The total number of individuals participating in the present study was 60. The mean age of participants was 47.13 years. Out of the 60 participants, 45 (75%) were male and 15 (25%) were female. Fifty-three participants (88.33%) were literate and seven (11.66%) were illiterate. A total of 49 (81.7%) were employed and 11 (18.3%) were unemployed, and 56 (99.33%) were married and four (6.66%) were unmarried (Table 1).

**Table 1:** Sociodemographic and clinical profile of the study population (N=60) *As per the Modified Kuppuswamy Socioeconomic scale

Parameter	Frequency (N=60)	Percentage (%)
Age Distribution		
21-30 Years	4	6.7%
31-40 Years	15	25.0%
41-50 Years	13	21.7%
51-60 Years	28	46.7%
Gender Distribution		
Male	45	75.0%
Female	15	25.0%
Literacy		
Literate	53	88.33%
Illiterate	7	11.66%
Occupation		
Employed	11	18.3%
Unemployed	49	81.7%
Socioeconomic Class*		
Lower	0	0%
Upper Lower	6	10.0%
Lower Middle	4	6.7%
Upper Middle	44	73.3%
Upper	6	10.0%
Marital Status		
Married	4	6.66%
Unmarried	56	93.33%
Covid Severity Category		
Mild	12	20.0%
Moderate	31	51.7%
Severe	17	28.3%
History	Yes	No
Family History of Comorbidity	15 (25.0%)	45 (75.0%)
Past Psychiatric Illness	0 (0.0%)	60 (100.0%)
Family History of Psychiatric Illness	0 (0.0%)	60 (100.0%)
Previous Hospitalisation	16 (26.7%)	44 (73.3%)
Smoking	14 (23.3%)	46 (76.7%)
Alcohol	11 (18.3%)	49 (81.7%)
Substance Abuse	0 (0.0%)	60 (100.0%)

As per the Modified Kuppuswamy Socioeconomic scale, six (10%) participants belonged to the upper lower class, four (6.7%) belonged to the lower middle class, 44 (73.3%) belonged to the upper middle class, six (10%) belonged to upper class, and none belonged to lower class in the present study population. Out of 60 participants, 12 (20%) belonged to the mild category, 31 (51.7%) belonged to the moderate category, and 17 (28.3%) belonged to the severe category as shown in Table 1.

Fifteen subjects (25%) had a family history of some comorbidity. None of the study participants reported a history of past psychiatric illness or any family history of psychiatric illness. Sixteen subjects (26.7%) reported a history of previous hospitalization, 14 (23.3%) had a history of smoking, and 11 (18.3%) had a history of alcohol consumption. None reported a history of substance abuse (Table 1). 

The most common complaint was fever reported by 55 (91.7%) individuals followed by shortness of breath reported by 53 (86.7%). Forty-seven (78.3%) subjects reported cough, 30 (50.0%) reported sore throat, 15 (25%) reported fatigue, 16 (26.7%) reported body ache, eight (13.3%) reported diarrhea, five (8.3%) reported a loss of smell, and 10 (16.7%) reported a loss of taste. 

Out of the 60 subjects participating in the present study, 29 (48.3%) reported having one or more pre-existing comorbidities. Eighteen (30.0%) had hypertension, followed by 16 (26.7%) with diabetes mellitus, eight (8.33%) with coronary artery disease, three (5%) with chronic obstructive pulmonary disease, and two (3.3%) with hypothyroidism.

The prevalence of depression, anxiety, and stress was checked on day 7 of hospital admission, on day 14, and on day 28 after discharge from the hospital. As we progressed from day 7 to day 28, a decline in the prevalence and severity of psychosocial manifestations was seen as shown in Table 2. 

**Table 2:** Prevalence of Depression, Anxiety, and Stress on Day 7 of admission, Day 14, and Day 28 after discharge from hospital (N=60) *P value < 0.05 is considered significant

Parameter	Severity	Absolute Number of Cases			P-value
		Day 7	Day 14	Day 28	
Depression	None	9	41	56	<0.001*
	Mild	20	13	4	
	Moderate	20	6	0	
	Severe	7	0	0	
	Extremely Severe	4	0	0	
Anxiety	None	9	41	56	<0.001*
	Mild	20	13	4	
	Moderate	20	6	0	
	Severe	7	0	0	
	Extremely Severe	4	0	0	
Stress	None	44	41	56	0.007*
	Mild	9	13	4	
	Moderate	7	6	0	
	Severe	0	0	0	
	Extremely Severe	0	0	0	

As we progressed from day 7 to day 28, an increasing trend in scores was seen for all four domains of the WHOQOL-Bref scale, which implies an increase in the quality of life of study subjects (Table 3).

**Table 3:** Comparison of WHOQOL-Bref (Hindi version) scores from day 7 to day 28 *P value < 0.05 is considered significant WHOQOL-Bref: World Health Organization Quality of Life Brief Version

Domain	Day after admission	Mean (SD)	p-value
Physical Domain	Day 7	66.23 (12.5)	0.001*
	Day 14	77.43 (11.72)	
	Day 28	82.18 (10.02)	
Psychological Domain	Day 7	73.93 (12.21)	0.001*
	Day 14	78.33 (9.96)	
	Day 28	86.21 (6.31)	
Social Domain	Day 7	82.63 (16.12)	0.001*
	Day 14	86.38 (11.1)	
	Day 28	89.73 (6.89)	
Environmental Domain	Day 7	78.33 (12.68)	0.001*
	Day 14	88.78 (8.09)	
	Day 28	90.98 (5.46)	

The mean D-dimer levels were 957.32 ± 650.91 (ng/ml). The mean PCT levels were 1.04 ± 1.47 (ng/mL). The mean ferritin levels were 722.24 ± 486.75 (µg/L). The mean CRP levels were 65.36 ± 35.12 (mg/L). The mean IL-6 levels were 62.79 ± 49.05 (pg/ml). The prevalence and severity of depression were significantly associated with inflammatory markers namely, D-dimer, CRP, ferritin, PCT, and IL-6 (p < 0.05) as shown in Table 4.

**Table 4:** Association of depression on the DASS-21 scale with inflammatory markers (N = 60) *P value < 0.05 is considered significant IL-6: interleukin-6, CRP: C-reactive protein; DASS-21: Depression, Anxiety, and Stress Scale, 21 items

Marker	Depression on DASS 21 Scale	Number of cases		p-value
		Marker normal	Marker raised	
D-Dimer (ng/ml)	None	6	16	0.009*
	Mild	0	17	
	Moderate	0	13	
	Severe	0	8	
Procalcitonin (ng/ml)	None	20	2	<0.001*
	Mild	2	15	
	Moderate	0	13	
	Severe	0	8	
Ferritin (ng/ml)	None	11	11	<0.001*
	Mild	0	17	
	Moderate	0	13	
	Severe	0	8	
CRP (mg/L)	None	21	1	<0.001*
	Mild	2	15	
	Moderate	0	13	
	Severe	0	8	
IL-6 (pg/ml)	None	21	1	<0.001*
	Mild	0	17	
	Moderate	0	13	
	Severe	0	8	

No significant association was seen between anxiety and markers like D-dimer and ferritin. No significant association was seen between inflammatory markers and the prevalence and severity of stress.

## Discussion

The number of participants belonging to disease severity categories of mild, moderate, and severe in the present study were 12 (20%), 31 (51.7%), and 17 (28.3%), respectively. The prevalence of mild, moderate, and severe disease in a study by Arshad et al. was found to be 51.26%, 15.13%, and 18.91%, respectively [11].

Hossain et al. estimated the prevalence of anxiety and depression in South Asian countries during the COVID-19 pandemic. The prevalence of depression was similar among males (36.7%) and females (37.8%). The prevalence of mild, moderate, and severe depression was 25.11%, 13.91%, and 11.97%, respectively [12]. A similar prevalence of depression was seen in the present study on day 7 of hospital admission; 17 (28.3%) subjects had mild depression, 13 (21.7%) had moderate depression, and eight (13.3%) were found to have severe depression. In a study done by Hossain et al., the pooled prevalence of anxiety was estimated to be 41.3% and that of depression was found to be 34.1% [12]. However, in the current study, the pooled prevalence of anxiety and depression was slightly higher which is around 85% for anxiety and 63.3% for depression.

Vahedian et al. estimated the prevalence of depression, anxiety, and stress as 54.29%, 97.29%, and 46.61%, respectively [13]. The prevalence of depression and anxiety in the current study was 63.3%, and 85%, respectively, which was comparable to the previous study. However, the prevalence of stress in the current study was 26.7%, which was lower. In Vahedian et al.'s study, the proportion of employed individuals was 52.1%, and unemployed were 47.9% [13]. In the current study, the proportion of employed individuals was 81.7% and unemployed individuals were 18.3%. The higher employment rate in the present study can be explained by the fact that the present study includes hospital-based data, which may not be a reflection of the general population. In Vahedian et al.'s study, the proportion of unmarried participants was 55.21% while that of married participants was 44.79% [13]. In the present study, the proportion of married and unmarried participants was 93.3% and 6.7%, respectively.

In Yadav et al.'s study of SARS-CoV-2 patients admitted to a rural tertiary care hospital, they concluded that 66% of patients had moderate depression, while 50% of patients had severe anxiety [14]. The high prevalence of depression and anxiety was attributed to financial loss, loss of lives of loved ones, and fear of loss of their own lives. The proportion o participants who had depression and anxiety in the current study was 63.3% and 85%, respectively. The higher prevalence of depression and anxiety in the current study could be due to differences in healthcare infrastructure between urban and rural populations.

Singh et al. reported the prevalence of depression as 38.4% in SARS-CoV-2 patients admitted to a tertiary care hospital. It was also seen that the prevalence of depression increased by eight times as the duration of hospital stay increased beyond five days [15]. In the present study, the prevalence of depression was 63.3%; however, no interrelation could be drawn between the duration of hospital stay and the prevalence of depression.

The current study concluded that the prevalence and severity of depression, anxiety, and stress decreased with the progression of time. The prevalence of depression on day 7 of admission was 63.3%, which decreased to 33.7% on day 14 and further to 6.7% on day 28 after discharge. The prevalence of anxiety decreased from 85% on day 7 to 31.7% on day 14 and further to 6.7% on day 28. Similar findings were seen in a study conducted by Parker et al. [16]. In their study, the prevalence of depression was 29% and that of anxiety was 36% initially. At two week follow-up, the prevalence of depression decreased to 25% and that of anxiety decreased to 9%. In the present study, the non-pharmacological intervention comprised specially tailored tele-counseling therapy sessions for COVID-19 patients which were carried out for all study subjects by an experienced psychiatrist. On days 14 and 28 of follow-up, none of the patients had clinically significant depressive or anxiety disorder that warranted pharmacological intervention. Depression and anxiety scores on objective assessment dropped down to zero and subsequent follow-up of post-discharge therapy sessions was continued on an outpatient basis by the Department of Psychiatry.

Ali et al. concluded that CRP levels were elevated in 86% of SARS-CoV-2 infected patients. Elevated levels of CRP were found to be associated with increased disease severity. The mean concentration of CRP in mild disease was about 23 mg/L and in severe disease was about 46 mg/L [17]. In the current study, the mean CRP levels were found to be 65.36 mg/L. The current study also showed a positive association between CRP levels and the severity of SARS-CoV-2 infection (p < 0.05). A significant association between increased CRP levels and the prevalence of depression (p < 0.001) and anxiety (p < 0.011) was also seen in the present study. Hamilton et al. found that patients who had higher baseline serum CRP concentrations had a 40% more chance of developing depression during the SARS-CoV-2 pandemic [18]. This finding was consistent with the current study in which a positive association was seen between the prevalence of depression and increased serum CRP levels (p < 0.001).

Guirao et al. concluded that increased serum levels of IL-6 (> 35 pg/ml) were associated with increased severity of SARS-CoV-2 pneumonia, need for ventilation, and increased mortality [19]. In the present study, the mean serum levels of IL-6 were found to be 62.79 ± 49.05 pg/ml. Also, a significant association was seen between increased levels of IL-6 and the prevalence of depression (p < 0.001) and anxiety (p < 0.049).

Liu et al. found that elevated levels of inflammatory markers like CRP, D-dimer, IL-6, and serum ferritin were associated with the severity of infection. High baseline levels of IL-6 were found to be associated with increased core body temperature, and increased levels of D-dimer, CRP, lactate dehydrogenase (LDH), and serum ferritin [20]. A positive association between the prevalence of depression, anxiety, and stress and increased levels of D-dimer, PCT, and serum ferritin was also seen in the present study (p < 0.001). Increased PCT levels were also associated with an increased prevalence of anxiety (p = 0.008).

Hawlader et al. assessed the quality of life in recovered SARS-CoV-2 patients. The mean scores of QoL for the physical, psychological, social, and environmental domains were found to be 68.25±14.45, 63.28±15.48, 65.10±15.78, 62.77±13.07, respectively [21]. In the present study, the domain scores for physical, psychological, social, and environmental domains on day 7 of admission were found to be 66.23 ± 12.51, 73.93 ± 12.22, 82.63 ± 16.12, and 78.33 ± 12.69, respectively. In Hawlader et al.'s study, scores of physical and psychological domains were found to be significantly lower among females than male participants (p<0.001) [21]. This finding was contradictory to our study in which domain scores were higher for females than male participants. This finding could be explained by the presence of fewer co-morbidities in female participants in the present study. The current work found the environmental domain score to be 76.62 ± 11.71 in males and 83.47 ± 14.50 in female participants (p = 0.035). In a study by Hawlader et al., the quality of life score among employed participants was found to be 1.8 times higher than among unemployed participants. Low quality of life score in Hawlader et al.'s study was associated with factors like the presence of chronic diseases, increasing age, and the need for hospital admission during SARS-CoV-2 infection. In that study, an increase in quality of life score was seen in all domains except the psychological domain [21]. Those findings of quality of life scores of Hawlader et al.'s study contrasted with the present study, in which an increase in all four domain scores was seen.

## Conclusions

The SARS-CoV-2 pandemic not only affected an individual clinically and physically but also affected the individual’s psychosocial well-being. The prevalence of depression, anxiety, and stress on day 7 of admission in our study population was found to be 63.3%, 85%, and 26.7%, respectively. We concluded that at the two-week and four-week follow-ups, the prevalence of depression, anxiety, and stress decreased in our study subjects. We also concluded that increased levels of inflammatory markers were associated with increased severity of SARS-CoV-2 infection and with the prevalence and severity of depression and anxiety among study subjects. It was concluded in our study that the WHOQOL-Bref score was low during admission to the hospital as compared with the score after discharge from the hospital. An increase in WHOQOL-Bref score in all four domains namely Physical, Psychological, Social, and Environmental Domain was observed at two-week and four-week follow-ups. This concludes an increase in the overall quality of life among the study population after discharge from the hospital.
